The article "Grammar enhancement in EFL instruction: a reflection on the effects of self-evaluation, teacher support, and L2 grit" was retracted in 2025. Reasons: a compromised editor; unreliable results or conclusions; concerns about the peer review; concerns about the citations.

# Grammar enhancement in EFL instruction: a reflection on the effects of self-evaluation, teacher support, and L2 grit

**DOI:** 10.1186/s40359-023-01504-9

**Published:** 2024-01-04

**Authors:** Kelu Wang

**Affiliations:** School of Foreign Languages, Leshan Normal University, 614000 Leshan, China

**Keywords:** Grammar Learning, Self-evaluation, Teacher support, L2 grit, EFL Learners

## Abstract

Advancement in learning grammar and using it practically is one of the challenges of English as foreign learners (EFL) learners. Its progression may be expedited or slowed down by a variety of causes. Among the crucial factors, the possible effects of self-evaluation, teacher support, and L2 grit were still untouched which is the target of the current research. In so doing, 86 EFL students at the intermediate level were divided into two groups (i.e., experimental group and control group). The students in the control group (CG) are exposed to normal education, whereas learners in experimental group (EG) get extra instruction to practice self-evaluation and L2 Grit. Moreover, the emphasis on the teacher’s position as a facilitator and supporter was more prominent in the EG. Based on data screening which was completed via one-way ANCOVA, learners in EG were more successful in grammar assessment due to the treatment. Further research avenues and educational implications were elaborated upon.

## Introduction

Engaging in self-evaluation activities have the capacity to adversely impact several aspects of learners’ lives, including their mental well-being, among other possible consequences. Moreover, [1] found a positive correlation between a high self-evaluation and improved emotional regulation and academic achievement in EFL students. The use of self-evaluation approaches enables students to develop critical thinking skills and decision-making abilities, hence enhancing their capability to effectively address classroom challenges [2]. Likewise, [3] underscored the potential of self-evaluation as a means to guide students towards cultivating preferred emotional states. Academic support includes the provision of beneficial literature, materials, and resources by the instructor to learners. On the other hand, personal and emotional support involves the teacher providing affective assistance, including empathy, trust, and care. In the context of an L2 classroom, instances of L2 teacher support may include both academic support, which pertains to learning-related help, and personal support, largely focused on emotional well-being [4]. When a language student has the encouragement and support of teachers, they are significantly more likely to stay excited and optimistic about their studies. They are also less inclined to quit up since the support of others around them may generate a sense of responsibility [5].

The article "Grammar enhancement in EFL instruction: a reflection on the effects of self-evaluation, teacher support, and L2 grit" was retracted in 2025. Reasons: a compromised editor; unreliable results or conclusions; concerns about the peer review; concerns about the citations.

The concept of grit may be delineated as a combination of diligent exertion, steadfastness, and an aspiration for enduring objectives shown by pupils. The findings of [6] indicate that individuals with a notable level of grit have a favorable outlook towards their occupational endeavors. When seen from an alternative standpoint, the characteristic of grit as a personal quality bestows individuals with the ability to focus their endeavors and engage in several endeavors in order to achieve their goals [7]. The concept of learner L2 grit was first introduced by [8], highlighting the significance of an individual’s unwavering dedication and enthusiasm in pursuing and achieving their desired objectives.

Effective instruction and evaluation require school administrators, curriculum developers, and individual teachers to address both the emotional and intellectual well-being of the students. Students need access to self-evaluate resources and methods of making informed choices in order to effectively overcome the challenges associated with acquiring a second or foreign language. EFL learners may significantly improve their English grammar skills by adopting a self-evaluation method, receiving guidance from teachers, and using L2 grit frameworks. Grammar is a linguistic framework that structures a language into coherent and comprehensive sentences. It has the ability to comprehend the way words and phrases combine together to form logical and meaningful expressions. Grammar enables individuals to accurately convey their thoughts and engage in effective communication with others by adhering to linguistic rules that ensure coherence and comprehensibility. It enables learners to articulate their thoughts with clarity and refine the intended meaning of their messages [8]. To get progress in English grammar, learners particularly EFL learners need their teachers’ support and other learner attributed constructs to foster their success [9]. Enhanced grammatical proficiency is not solely critical for facilitating effective discourse, but also for cultivating a favorable reputation in academic and professional environments [10].

With regard to the extant research, the reciprocal interaction between these notions occurred in complete darkness. The findings of this research have the potential to be valuable in both the theoretical and practical domains. It is likely that it will further improve the understanding and consciousness related to online language instruction and evaluation, hence ensuring effective language acquisition. Considering these perspectives, the following study question and null hypothesis were formulated:

The article "Grammar enhancement in EFL instruction: a reflection on the effects of self-evaluation, teacher support, and L2 grit" was retracted in 2025. Reasons: a compromised editor; unreliable results or conclusions; concerns about the peer review; concerns about the citations.

### RQ

Do self-evaluation, teacher support, and L2 grit enhance English grammar learning?

### HO

Self-evaluation, teacher support, and L2 grit do not enhance English grammar learning.

## Literature review

### Self-evaluation

Assessment serves as a systematic basis for drawing inferences regarding the progress of students’ growth and their acquisition of knowledge. Over time, several methodologies have been developed to streamline the assessment process and improve its credibility and consistency. self-evaluation is a method of evaluation in which learners actively participate in assessing their own behaviors, attitudes, or performance. It is essential to foster an environment that promotes and provides training for each learner to take part in the self-assessment process [11]. Similarly, [12] posits that the fundamental concepts of self-evaluation include critical thinking, metacognition, monitoring, and self-regulated learning. Moreover, the study conducted by [13] has classified as a higher-order quality that encompasses several psychological constructs such as self-esteem, generalized self-efficacy, neuroticism, and locus of control. According to [14], students who engage in processes acquire the ability to engage in comprehensive thinking and make informed decisions. Additionally, these students may develop improved strategies for coping with academic challenges.

The use of strategies in self-assessment in online education facilitates learners’ awareness and monitoring of their own learning progress. The effects of engaging in self-evaluation extend beyond cognitive development, as learners’ emotional well-being is also affected by the approaches used. Additionally, it was emphasized that EFL students who possess elevated levels of self-awareness may exhibit enhanced emotional regulation skills and demonstrate greater proficiency in acquiring language skills [15]. This implies that the implementation and use of self-evaluation practices have an impact on the cognitive, metacognitive, and emotional aspects of students’ academic experiences [16]. Additionally, it has been shown that several elements have the potential to establish the tone of student-teacher interaction among learners. Furthermore, [17] conducted studies that examined the impact of emotion management, buoyancy, and reflection on learners’ accomplishment in self-evaluation and their ability to manage test taking in online assessments.

### Teacher support

The concept of “teacher support” encompasses a wide range of assistance, guidance, and camaraderie provided by the educator [18] argue that academic aid and personal/emotional support are integral aspects of it. The provision of personal and emotional support by teachers includes the provision of affective support, including but not limited to empathy, trust, and care, as outlined by [19]. As defined by [20], academic support pertains to the instructional endeavors aimed at facilitating the acquisition of knowledge and skills by students. On the other hand, emotional support encompasses the learners’ experience of affection, admiration, and care from the teacher throughout the learning journey.

The article "Grammar enhancement in EFL instruction: a reflection on the effects of self-evaluation, teacher support, and L2 grit" was retracted in 2025. Reasons: a compromised editor; unreliable results or conclusions; concerns about the peer review; concerns about the citations.

The literature indicates a correlation between the provision of support by second language (L2) teachers and various outcomes for second language learners. Specifically, [21] found a relationship between L2 teacher support and learner engagement, while [22] demonstrated a connection between L2 teacher support and learner achievement. Additionally, [4] established a link between L2 teacher support and positive academic affect in second language learning. Moreover, previous research has shown that the provision of support from second language (L2) teachers has a significant role in enhancing the enjoyment experienced by learners in foreign language classrooms. This is achieved by fostering a sense of appreciation among L2 learners towards their instructors [21]. This sense of appreciation contributes to an enhanced level of satisfaction in foreign language courses. In a recent study conducted by [23], it was shown that students with lower abilities demonstrated enhanced English language learning when they received substantial support from their teachers. This discovery underscores the positive impact of teacher assistance on student achievement.

 [24] propose that the provision of support by instructors is an additional crucial element in enhancing students’ behavioral engagement within educational settings [25] discovered a favorable correlation between teacher support and behavioral engagement. Moreover, it was shown that the relationship between teacher support and social, emotional, and cognitive engagement was mediated by behavioral engagement [1] conducted research indicating that the influence of instructors on students’ academic achievement is contingent upon the degrees of motivation shown by the students. According to a longitudinal study done by [26], it was seen that the provision of teacher assistance had a significant and positive influence on the self-efficacy and motivation of adolescent students. According to [21], teacher support emerges as a robust and reliable predictor of motivation, exerting a significant influence on the motivated learning behavior of L2 learners. The concept of grit has a robust correlation with the construct of motivation. The goal-oriented nature of L2 grit aligns with the concept of directed motivational current, as outlined in the study conducted by [27].

The article "Grammar enhancement in EFL instruction: a reflection on the effects of self-evaluation, teacher support, and L2 grit" was retracted in 2025. Reasons: a compromised editor; unreliable results or conclusions; concerns about the peer review; concerns about the citations.

### L2 grit

The notion of grit pertains to the act of exerting significant effort in the face of adversities, persisting in one’s endeavors and sustaining interest for an extended period of time, even in the presence of setbacks, adversity, and periods of stagnant growth [11, 28] posited that, in addition to ability, tenacity plays a significant role in the academic success of learners. The concept of L2 grit in learning was introduced by [11, 29], who emphasized the importance of people’ enthusiasm and relentless efforts in pursuing their own goals. Enthusiasm pertains to the heightened level of enthusiasm and motivation shown by people in their pursuit of a certain objective. According to [30], perseverance is a crucial component of grit that motivates people to fully dedicate themselves to the many stages involved in pursuing a certain objective. In the work of [31], the authors claim that grit is a quality that is distinctive to certain domains. In light of this characteristic of grit, [32] developed and verified a measurement tool called “the Language-domain-specific grit” in order to evaluate the level of grit shown in language courses.

As stated by [33], students who possess a higher level of grit have increased levels of enthusiasm and dedicate more time to their educational pursuits. Specifically, those who possess elevated levels of grit have a propensity to persist in pursuing their long-term objectives despite encountering challenges and obstacles [30–32]. In the words of [11], the presence of grit in learners enables them to effectively manage stress and anxiety, resulting in favorable dispositions towards work-related matters and active engagement. In light of its significance and endorsement in enhancing personal welfare, several educational organizations have endeavored to design, implement, and execute instructional materials and syllabi that include the concept of grit into their educational curricula [27].

The examination of the scholarly literature on learner grit reflects the prevailing focus on the reciprocal relationship between students’ grit and its expressions within the academic domain. An example of this may be seen in the study conducted by [34], where they established a positive correlation between L2 grit and achievement in the English language. Furthermore, [35] has provided further evidence to support the notion that EFL students’ academic desire and growth mindsets have a mediating role in their level of grit. Similarly, the study conducted by [36] shown that proficient management of emotions positively influences the L2 perseverance, emotional regulation (ER), and resilience of EFL learners. Therefore, it can be inferred that the combination of L2 grit and a harmonious psychological condition among students significantly impact the whole language development process.

The article "Grammar enhancement in EFL instruction: a reflection on the effects of self-evaluation, teacher support, and L2 grit" was retracted in 2025. Reasons: a compromised editor; unreliable results or conclusions; concerns about the peer review; concerns about the citations.

## Method

### Settings and participants

A sample of 86 students from a private language institute in China participated in this study. The students in this group were chosen after taking the Oxford Quick Placement Test. This study was designed for students whose English proficiency is at the intermediate level. During the course of this work, no more English instruction was allowed. Students ranged in age from 14 to 16; there were 41 females and 45 males. The research does not take into account the subjects’ sociocultural background. They have 16 sessions to complete their program and pass. Students gave their informed consent to participate in this study, and their participation was completely voluntary.

### Materials

The Oxford Quick Placement Test (OQPT) was given in order to assess the English language skills of the students. The OQPT utilizes a score range of 0.1 to 0.9. Within this range, scores falling between 0.4 and 0.6 are designated as indicative of an intermediate level of skill in the English language. The research found that the reliability coefficient of the OQPT was 0.91.

Based on the contents of the proposed resources, a researcher-created exam with 50 items was developed (Understanding and Using English Grammar). In doing so, three psychometricians and three EFL teachers were asked to assess the item quality. Some elements were altered in response to their feedback. Following this, the test was administered to a group of 42 EFL students similar of the target demographic to assess test-retest reliability. The identical examination was re-administered to the same subject after 1 month to assess the stability of the findings across time. According to the Pearson correlation coefficients, the test has a significant test-retest reliability (r = .85).

The self-evaluation of the participants was measured with the (CSEQ), which was devised and validated by [37]. This 5-point Likert scale consists of 12 questions with the following response options: strongly disagree (1) and strongly agree (5). On this scale, scores varied between 12 and 60. On this scale, high scores indicated positive self-evaluation, whereas low scores indicated negative self-evaluation. In the current investigation, CSEQ’s reliability was 0.873, indicating an acceptable Reliability.

The Teacher Support Measure (TSM) developed by [19] was used to evaluate TS. The measure consisted of eight questions divided into two scales: teacher academic support and teacher personal support. On a 5-point Likert scale, respondents may choose between always (1) and never (5). English was added to the scale’s question wording so that it could be used to assess teachers’ ability to provide help in a particular subject area.

The article "Grammar enhancement in EFL instruction: a reflection on the effects of self-evaluation, teacher support, and L2 grit" was retracted in 2025. Reasons: a compromised editor; unreliable results or conclusions; concerns about the peer review; concerns about the citations.

The Language‑domain‑specific Grit Scale (LDSGS) developed and validated by [32] was used to evaluate the fortitude of EFL university students. This scale consists of 12 items, six of which assess perseverance of effort and six of which assess consistency of interest on a five-point Likert scale ranging from 1 “not at all like me” to 5 “very much like me.” In this examination, the reliability of the (L2-Grit) as determined by Cronbach’s alpha (ranging from 0.818 to 0.879) was noteworthy.

### Procedures

The present research utilized a quasi-experimental design in the first phase, and individuals were randomized to groups based on non-random factors. Initially, the Oxford Quick Placement Test was utilized to measure the level of English language competency of the students. 86 participants were selected for the current research based on the results of the Oxford Quick Placement Test (score range 0.1–0.9) and the cut score (0.4–0.6). Students with higher scores (between 0.7 and 0.9) indicating high language competence were excluded, whereas students with intermediate English language competency were invited to participate in this research.

Following the pre-test, training was provided the researcher, who taught all of the courses in both the EG (n = 42) and CG (n = 44). This research was conducted over the course of one semester (16 sessions) in 2023. The material applied in this study was Understanding and Using English Grammar by [38]. This book was used for both groups to learn English grammar. The participants engaged in virtual instruction via the use of Tencent Meeting. Additionally, a private group was established on the messaging platform WhatsApp, whereby the researcher of this study shared textual content aimed at offering solutions for the enhancement of self-evaluation and L2 grit. These techniques are derived from the pertinent literature and relevant scholarly sources. In the event of encountering difficulties, individuals may choose to communicate by telephone. Students may pose their inquiries and the instructor will provide the necessary feedback. Additionally, learners’ homework was checked by the teacher.

English learners were also urged to maintain a notebook and evaluate their own grammar learning experiences and report their reflections as well as their progress to their teachers. Within the context of this What’s App group, EFL students in EG engaged in collaborative exercises either in pairs or small groups, with a strong emphasis placed on fostering social connections and providing mutual support. It is worth noting that the instructors of both groups are the same. In session 16, before to the final assessment of the participants, a post-test was administered to both the CG and EG. This post-test aimed to evaluate the development of English grammar and determine the effectiveness of the project. The post-test included measures of English grammar, self-evaluation, teacher support, and L2 grit. Both the pre- and post-tests were administered in English since the subjects were competent enough to complete the scales in that language. The validation of the reliability of the findings was conducted by three EFL instructors via the administration of pre- and post-tests.

The article "Grammar enhancement in EFL instruction: a reflection on the effects of self-evaluation, teacher support, and L2 grit" was retracted in 2025. Reasons: a compromised editor; unreliable results or conclusions; concerns about the peer review; concerns about the citations.

### Data analysis

A one-way ANCOVA was conducted to examine the effectiveness of self-evaluation, teacher support, and L2 grit in grammar enhancement in EFL instruction. Prior to doing one-way ANCOVA, many underlying assumptions were assessed, including normality, sample size, outliers, linearity, and homogeneity of regression. ANCOVA examines the impact of a covariate variable on the variance of the dependent variable and distinguishes it from the variance changes caused by variations in the levels of a qualitative variable. As a result, it reduces the uncertain fluctuations in the dependent variable’s variance (error) and produces more accurate outcomes [39].

## Results

Firstly, the normality of the distribution was checked via Kolmogorov-Smirnov (KS) and the results of which are indicated in Table 1:

**Table 1:** Kolmogorov-Smirnov results for the English grammar pretest and posttest of both groups

	Statistic	df	Sig.
EG English Grammar Pre	0.069	42	0.200
EG English Grammar Post	0.146	42	0.075
CG English Grammar Pre	0.155	42	0.093
CG English Grammar Post	0.118	42	0.155

The *Sig.* value under the KS part of the table represented a value higher than 0.05, which indicates that the distribution of scores was normal. Thus, it is logical to run independent samples t test and one-way ANCOVA.

**Table 2:** Descriptive statistics for comparing pretest scores of the EG and CG

	Groups	N	Mean	Std. Deviation	Std. Error Mean
English Grammar Pretest	EG	42	27.2857	7.73111	1.19294
	CG	44	28.8864	8.55955	1.29040

It could be seen in Table 2 that the difference between the EG (*M* = 27.2857) and CG (*M* = 28.8864) mean scores on the pretest of English grammar was quite small. In order to find out whether this difference between the pretest scores of both groups was statistically significant or not, the following *t* test needs to be considered:

The article "Grammar enhancement in EFL instruction: a reflection on the effects of self-evaluation, teacher support, and L2 grit" was retracted in 2025. Reasons: a compromised editor; unreliable results or conclusions; concerns about the peer review; concerns about the citations.

**Table 3:** Independent-samples t test comparing the pretest of EG and CG

		Levene’s Test for Equality of Variances		t-test for Equality of Means				
		F	Sig.	t	df	Sig. (2-tailed)	Mean Difference	Std. Error Difference
English Grammar Pretest	Equal variances assumed	1.474	0.228	− 0.909	84	0.366	-1.60065	1.76154
	Equal variances not assumed			− 0.911	83.751	0.365	-1.60065	1.75734

Based on Table 3., there was not a statistically significant difference in the pretest scores for EG and CG, as *p* = .366 (two-tailed). Hence, it could be inferred that the learners in the two groups were at the same level of grammar before the treatment.

As the vital research question of the study was intended to figure out whether self-evaluation, teacher support, and L2 grit enhance English grammar learning, the posttest scores of the EG and CG learners were compared. To attain this objective, one-way ANCOVA was run:

**Table 4:** Descriptive statistics for comparing the post-test scores of the EG and CG

Groups	Mean	Std. Deviation	N
EG	38.9524	6.13249	42
CG	32.6364	7.67385	44
Total	35.7209	7.61678	86

In Table 4, the post-test mean score of the EG (*M* = 38.9524) was higher than the posttest mean score of the CG (*M* = 32.6364). To find out whether this difference was a statistically significant one or not, the *Sig.* column in Table 5 must be checked:

**Table 5:** Results of one-Way ANCOVA for comparing the post-test scores of the EG and CG

Source	Type III Sum of Squares	df	Mean Square	F	Sig.	Partial Eta Squared
Corrected Model	3174.62	2	1587.314	74.99	0.000	0.64
Intercept	2061.37	1	2061.376	97.39	0.000	0.54
English Grammar Pre	2317.41	1	2317.412	109.49	0.000	0.56
Groups	1148.18	1	1148.183	54.25	0.000	0.39
Error	1756.67	83	21.165			
Total	114666.00	86				
Corrected Total	4931.30	85				

In Table 5, the *p* value is lower than the alpha level of significance (i.e., p < .05) which shows that the difference between the two groups of EG and CG on the grammar posttest was statistically significant. This means that using the self-evaluation, teacher support, and L2 grit could significantly improve the grammar learning of the EG learners. Another important data in Table 5 is the Partial Eta Squared which equaled 0.39, which means that the treatment accounted for 39% of the difference between the EG and CG learners. The existence of a significant difference between the grammar post-test scores of the EG and CG learners is graphically represented in Fig. 1 below:

**Fig. 1:** Posttest Mean Scores of the EG and CG Learners

Figure 1 shows that the EG learners considerably outperformed the CG learners on the grammar posttest, indicating that the *treatment* had significant effects on Chinese EFL learners’ grammar learning.

The article "Grammar enhancement in EFL instruction: a reflection on the effects of self-evaluation, teacher support, and L2 grit" was retracted in 2025. Reasons: a compromised editor; unreliable results or conclusions; concerns about the peer review; concerns about the citations.

## Discussion

The goal of this study was to investigate the ways in which self-evaluation, support from teachers, and grit in learning a second language all influence the acquisition of English grammar via the medium of virtual language training. To achieve this goal, quasi-experimental study was conducted in China’s EFL training. The findings of ANCOVA demonstrated that EFL learners have the potential to enhance their grammar learning provided they acquire adequate levels of self-evaluation, teacher support, and L2 grit. As a result, the null hypothesis is not supported. This conclusion should not come as a surprise since it is well known that the elements that EFL students confront in online teaching and evaluation have an influence on the levels of anxiety that they experience if they are exposed to them. It is common for students to either not have any anxiety at all or to experience a large reduction in the intensity of their anxiety when they feel comfortable and encouraged by their professors to do their coursework.

It was discovered that self-evaluation acts as a mediator between the learners and their linguistic worries. This study found that the more self-reflective an EFL student is, the less disengaged they were about learning English grammar. It is determined that students, via the lens of self-evaluation, do extensive self-monitoring and evaluation for learning grammar. Higher-order thinking skills, a sense of self-worth, and learner confidence may be required to successfully complete this evaluation. According to [40–42], trainees will experience anxiety if they set goals that exceed their abilities. Therefore, EFL students need to be well-equipped with self-assessment strategies for dealing with negative emotions like nervousness in the classroom. To put it another way, the more EFL students practice self-evaluation, the more they learn about their own traits and values. The findings of [16, 18] are supported by the findings presented here. They were able to show that self-evaluation beliefs, cognitive abilities, self-regulatory mechanisms, and resilience are all closely connected to one another.

The manner in which students engage in self-evaluation has a role in shaping and reshaping a positive self-concept and self-identity, ultimately fostering the pursuit of worthwhile objectives. EFL students get advantages from such experiences as they aid in fostering an inherent sense of control and a perception of effectiveness in their ability to do tasks proficiently. The study’s findings underscore the importance of involving students in self-evaluation, as it motivates them to articulate the reasons and objectives behind their successful outcomes in terms of enhancing their proficiency and effort in mastering grammar structure. The profound effects of self-evaluation on language learning have been extensively examined via many theoretical frameworks and empirical studies on self-evaluation (e.g.,). Based on the Self-Determination theory [43], enhancing self-awareness results in an increase in educational aspirations, academic contentment, determination, and engagement in the classroom.

The article "Grammar enhancement in EFL instruction: a reflection on the effects of self-evaluation, teacher support, and L2 grit" was retracted in 2025. Reasons: a compromised editor; unreliable results or conclusions; concerns about the peer review; concerns about the citations.

Greater advancements in EG in the acquisition of grammatical skills, along with a heightened perception of teacher support, indicate that students who get sufficient and timely assistance from their English educators are more inclined to be motivated in their language studies and have a more favorable overall learning experience. The results also provide theoretical support to the control-value theory [44] on the linkage between feelings of achievement and their preceding factors in the context of second language learning. Prior studies in the field of language learning have largely overlooked the influence of teacher support on students’ negative perceptions of achievement [42, 45]. Further investigation on the relationship between teacher support and the reduction of other negative emotions is recommended.

To put it another way, students’ feelings of accomplishment may be directly and indirectly influenced by the perceptions they have of their teachers’ levels of support for them in their academic pursuits. A study conducted by [46] came to similar conclusions. The researcher discovered that students’ views of teacher support might either directly impact their academic engagement or indirectly influence it by altering the pleasure they took from studying arithmetic. To be more precise, students’ academic motivation, a key result of accomplishment emotions, may be affected by their perceptions of their teachers’ support in the classroom. Based on these results, control-value theory may be more broadly applied to the field of second language acquisition [47]. Teachers are encouraged to take steps including demonstrating keen interest in their students’ progress, providing analytical input, and employing a wide variety of instructional techniques to aid their pupils in their studies because teacher support is linked to students’ feelings of accomplishment and their level of academic engagement [48].

More specifically, the findings demonstrated that L2 grit has the ability to assist students in managing their anxiety around communication, fear of receiving a poor evaluation, anxiety regarding taking tests online, and anxiety related to taking classes in foreign languages. The results of a prior study, although a limited one, that indicated the significant role that grit plays in the control of emotions [49] confirm this conclusion, which is in agreement with the findings of the previous study. In the context of EFL, the results of [3] provided more evidence for the very important function that L2 grit plays in lowering the level of anxiousness experienced by learners and enhancing their general well-being during language evaluation. Additionally, [50] demonstrated that in the context of the argumentative task, both the persistence of effort and working memory play a significant role in determining how well a person does while writing in a second language (L2).

The article "Grammar enhancement in EFL instruction: a reflection on the effects of self-evaluation, teacher support, and L2 grit" was retracted in 2025. Reasons: a compromised editor; unreliable results or conclusions; concerns about the peer review; concerns about the citations.

In addition, it is possible to draw the conclusion that language students who have a greater degree of persistence and resilience are more likely to display persistent efforts in the pursuit of their particular goals. The degree to which people are able to retain consistency in their undertakings and aims has a direct influence on their capacity to evaluate their own growth and success. Validation of the connections between L2 grit and self-efficacy was accomplished within the same line of study [51]. When it came to self-evaluation, one of the most important ideas was self-efficacy. The results that [52] uncovered provided more evidence in support of this previous conclusion. The researcher arrived at the conclusion that the coping strategies used by learners were a reliable indicator of their capabilities in the area of self-evaluation. In the case of EFL, the result of [40] was also another piece of data that supported the critical role that L2 grit plays in increasing learners’ motivation to communicate in the target language.

## Conclusion

The results of the research have certain educational repercussions that might be drawn from them. The integration of psychological and mental aspects into the curriculum has the potential to enhance students’ accessibility to course materials. This is because the rapid proliferation of technological advancements and the increasing demand for online and virtual educational platforms have made it possible for students to access knowledge whenever it is convenient for them and from any geographical location, even outside of the confines of the traditional classroom setting. In light of this, teachers need to acquire the skills necessary to demonstrate digital literacy in order to make successful use of technological platforms for language education and assessment. To reiterate what was said before, it is of the utmost importance to foster a healthy psychological outlook in students throughout their whole educational experience. Within this framework, it is essential for both educators and students to have a comprehension of the notions of self-help and the possible influence that these concepts may have on the psychological and physiological well-being of the individuals involved.

The article "Grammar enhancement in EFL instruction: a reflection on the effects of self-evaluation, teacher support, and L2 grit" was retracted in 2025. Reasons: a compromised editor; unreliable results or conclusions; concerns about the peer review; concerns about the citations.

Grammar may be likened to a game. Those students who possess a deep understanding of the language acquire grammatical skills by intuitive means, while others have difficulties with aspects such as tenses, phrases, and sentences. The learners’ growth in grammar is fostered by instructors who are supportive, particularly in situations when the learners want assistance and feedback. Enhancing English grammar skills also includes engaging in writing exercises during class and pursuing personal writing endeavors outside of class for pleasure. An effective method to enhance writing skills is to engage in English discussions and responses in Instagram, Facebook, or Twitter updates in English. It is possible for instructors to assist their students in developing a strong foundation in English grammar by providing them with understandable explanations, relevant exercise, and consistent reinforcement. Thereby, it is important for teachers to modify their teaching methods in accordance with the requirements, interests, and various learning styles of their students.

The findings of the present study should be assessed considering the inherent constraints of empirical investigation. This study used a quasi-experimental technique, which featured intact groups that were included in the sample processes. Future research should use a variety of approaches to enhance the results of the current study. Furthermore, it is important to acknowledge that the sample sizes of the EG and CG were rather small, which might possibly affect the capacity to apply the results to a larger population. Subsequent investigations should use a more extensive sample size in order to provide more comprehensive analyses. The present research was also limited in its focus on the linguistic proficiency of students enrolled at an intermediate level of education. Subsequent investigations might potentially delve into supplementary areas of inquiry. Furthermore, this research examines the participants’ advancement in grammar. Subsequent research endeavors might explore other language competencies and assess the learners’ advancement in self-assessment, instructor assistance, and second language perseverance. Lastly, this research did not examine the potential effects of the demographic characteristics of the participants and their socio-cultural diversity, which can be the focus of future research.

The article "Grammar enhancement in EFL instruction: a reflection on the effects of self-evaluation, teacher support, and L2 grit" was retracted in 2025. Reasons: a compromised editor; unreliable results or conclusions; concerns about the peer review; concerns about the citations.

## Data Availability

No datasets were generated or analysed during the current study.

## Data Availability

The dataset of the present study is available upon request from the corresponding author.
